# Optimization of Vocal Singing Training Methods Using Intelligent Big Data Technology

**DOI:** 10.1155/2022/8589517

**Published:** 2022-07-09

**Authors:** Yong Lin, Kang Mao

**Affiliations:** ^1^Conservatory of Music, Jeonbuk National University, Jeonju 561756, Republic of Korea; ^2^Conservatory of Music, Huaiyin Normal University, Jiangsu 223300, China

## Abstract

The development of art education and information technology has led to the importance of computer technology and multimedia technology in the development of students' independent inquiry and research skills. In the context of “Internet+,” new modes of teaching phonics have emerged, reconfiguring the spatial and temporal relationship of phonics education. The use of Internet resources is not only a simple collection and sharing of educational resources, but also a new way of teaching voice, which has the magic charm of becoming one of the resources for the majority of voice enthusiasts. However, in practice, there are very few assistive software suitable for music classroom teaching. It is important to research and implement teaching aids suitable for music classroom teaching. Based on intelligent big data technology to optimize the phonetic training methods, the teaching methods are more specific, scientific, and diverse, and improve the self-learning ability and learning interest of Chinese phonetic learners. The experimental results show that the weight of the phonetic teaching optimization process is 0.154 higher than the weight before processing, which is expressed as the value of the control reliability fuzzy quantifier in this test. In other words, the reliability is “absolutely reliable.” Therefore, this study is expected to promote the modernization and scientific process of Chinese vocal education and propose a new way of thinking for Chinese vocal education.

## 1. Introduction

With the rapid development of the economy, music education in the Internet era is gradually developing in the direction of intelligence and networking [1]. Being in the new media environment is like being in a “university without walls.” New media has brought great convenience and development to modern education [2]. The biggest difference between vocal education and other education is that the vocal teaching method is relatively abstract with the focus on performance, and it is an art form that resonates directly with the subject matter [3], which can be concretized, visualized, and informed if intelligent big data technology is applied to the vocal teaching method [4]. A set of basic information management, student music assignment management, music practice management, online classroom management, and information notification management is built by making full use of web technology and combining the characteristics of music majors [5]. The integrated educational platform of student big data platform can develop students' potential more effectively, promote students to acquire learning skills, and improve learning efficiency [6].

Computer technology is increasingly infiltrating the field of education [7], thanks to its advantages of speed, efficiency, convenience, and wide connectivity. The development of society is dependent on “Internet+,” which allows us to innovate boldly [8]. It has enabled closer integration between industries for the benefit of society, increased people's convenience, and accelerated China's economic development [9]. Existing teaching methods have a number of flaws, including single teaching methods, a lack of teaching resources, and dull content, all of which are undergoing qualitative changes as computers are introduced [10]. In the future development of education and teaching, digitalization and informatization will become an unavoidable trend [11]. Vocal music is a highly technical and practical professional field [12]. It is both a science and an art. Learning by relying solely on theoretical knowledge and book materials is extremely difficult [13]. Correct vocal conditions, long and continuous hard training, and the singer's skills are all important factors in the vocal and singing process of vocal singing.

The use of intelligent big data technology to optimize vocal songs is undeniably of practical significance when traditional vocal music education is combined with information technology. In the traditional teaching process, live vocal music teaching solves the problems of uneven teacher distribution, timely teacher-student interaction during the teaching process, and passive student feedback after class [14, 15]. The following are the paper's unique features. (1) Using intelligent big data technology, an in-depth study and research on the teaching mode of vocal singing training are conducted, highlighting the benefits and drawbacks of the teaching mode and teaching form of vocal singing training. It also gives more room for future training methods to be improved. (2) This paper can analyze all of the students in a group specified by the teacher, such as several classes or a specific college, using a rule-based expert system, so that this system can better serve for teaching. (3) The purpose of this paper is to provide a systematic and comprehensive discussion and summary of vocal music teaching in the new media environment, including its uncertainty reasoning and optimization process.

## 2. Related Work

### 2.1. Vocal Music Training Method

In recent years, with the education goal of cultivating well-rounded and high-quality talents in the new era of China, music teaching, as an important part of quality education, has received the attention and love of many students. Whether for the love of the profession or for future employment, the number of students choosing music majors is increasing year by year, so colleges and universities have also taken this opportunity to expand their professional enrollment. With the help of the Internet platform and advantageous resources, a variety of innovative models such as massive open online courses, cell phone APPs, and WeChat have also emerged in vocal music teaching, which has laid a certain foundation for the development and research of vocal music teaching.

Medeiros et al. introduced the concept of e-learning support systems, the idea of which has been used until today. Under the influence of this idea, many similar e-learning service systems have been developed by foreign educational institutions and software manufacturers in the past two decades [16]. E-Learning support systems were proposed by Baker and Cohen et al., and their ideas have been used until today. Under the influence of this idea, many similar e-learning service systems have been developed by foreign educational institutions and software manufacturers one after another. The basic design model is to fully utilize computer multimedia technology to deliver knowledge to learners through video and audio [17]. Xiong et al. argue that the creation and development of the online classroom are based on the Internet. This Internet breaks the limitations of the traditional time and space processes, allowing learners to leave home and no longer be restricted by geography and time [18]. Li proposed three centers that represent “progressive education” in the traditional educational center of Herbart: the center of the teacher, the center of the classroom, the center of systematic book knowledge, the center of the child, the center of activities, and the center of personal direct marketing [19]. Chi argues that the emergence of online classrooms means that the walls of traditional campuses will be broken down and the traditional function of sharing quality educational resources will become inevitable [20].

After the informationization of music teaching resources, with the help of computer technology and the Internet, teaching resources are rapidly spread in the network, which will make it more convenient for students to obtain music teaching resources and knowledge, and learning will no longer be affected by geography and time.

### 2.2. Intelligent Big Data Technology

With the increasing number of students in colleges and universities, the teacher-student ratio has increased substantially compared to the past. In the limited teaching time, teachers pay more attention to the teaching of vocal expertise and some singing skills, making vocal teaching more theoretical. Big data technology is an emerging edge discipline developed on the basis of the interpenetration of computer science, cybernetics, information theory, neurophysiology, psychology, philosophy, linguistics, and other disciplines.

Yang proposed the Online Education Platform System, a representative online education platform that actively uses e-books and textbooks and has more than 100 million registered users [21]. Rosenzweig et al. describe the “Internet + education” model and propose that the “Internet + education” model should evolve into the “Internet education” model [22]. Simones and Lima concluded that although online voice teaching has many advantages over traditional voice teaching, it does not replace traditional voice in terms of the specificity of vocal music. Voice instruction is a teaching method. Sun pointed out that the education industry is facing the challenges of the “Internet+” era and the responsibility system of education informatization construction, and it is necessary to establish a “big database” in colleges and universities [23]. Sun pointed out that the education industry is facing the challenges of the “Internet+” era and the accountability of education informatization construction, and it is necessary to establish a “big database” for team analysis in universities [24]. “The concept of educational system proposed by Sturtevant can provide tools that allow even nontechnical general teachers to easily create online courses and secure websites for courses, homepages, student management, and learning process tracking functions” [25].

Therefore, through intelligent big data technology, learners can complete real-time playback of online learning resources within limited bandwidth without having to completely download courseware and learning materials. Learners can independently select a certain segment of learning content, and learning is more actionable and convenient.

## 3. Optimization of Vocal Singing Training Method Based on Intelligent Big Data Technology

### 3.1. Big Data Technology Optimizes Vocal Training and Establishes Expert System

The combination of big data technology and music has existed for quite a long time, the development of digital sound processing and software programs for music has made great progress, and the combination of big data technology and music education has produced numerous research results [26]. Vocal teaching can be divided into two parts: vocal practice and song singing, and vocal practice is the basis of song singing, so it is very important to practice vocal practice [27]. With the help of multimedia and the development of emotional robots and deep learning, the efficiency of learning and practicing is greatly improved and a good training cycle will be formed, as shown in Figure 1.

To begin with, the teacher's explanation of vocal exercises in the traditional vocal teaching mode is very abstract. Only the student's own understanding and comprehension can cause him or her to feel it. Students can intuitively feel the application and changes of the diaphragm, throat, mouth, tongue, teeth, and other organs and grasp their rules by showing 3D animations of concepts such as “breathing” and “resonance” in the process of introducing modern information technology into vocal teaching. The content of vocal teaching for acting training is usually chosen by the teacher, who uses models to sing and explain the work, so catering to the acceptance of all students will inevitably be difficult. The best student in the current class is the teacher, because he or she is the one who knows the most. The following formula calculates the difference between the current average student level and the corresponding teacher level for each subject:

(1) $$\begin{array}{c} \text{Difference}-{\text{Mean}}_{j,}i=r_{i}\left(X_{j,k\text{best},i}-\text{TF}\times M_{j,i}\right). \end{array}$$

*X*_*j*,*k*best,*i*_ is teacher's level in subject *j*.

*r*_*i*_ is random number from 0 to 1.

TF is teaching factor.

TF is randomly determined as 2 or 3 by the following formula:

(2) $$\begin{array}{c} \text{TF}=\text{round}\left[2+\text{rand}\left(0,1\right)\right]. \end{array}$$

Therefore, to build an expert system, the development process follows the same steps and principles of software engineering as any other large software development process. The development toward emotional robotics and deep learning [28] with the help of multimedia significantly increases the efficiency of learning and practice. The process of the student phase is to adjust the learning by analyzing the differences between the two students. The stage process is shown in the following equation:

(3) $$\begin{array}{c} X_{j,P_{i}}^{\prime }=\left\{\begin{array}{cc} X_{j,P_{i}}^{\prime }+r_{i}\left(X_{j,P_{i}}^{\prime }-X_{j,Q_{i}}^{\prime }\right), & f\left(X_{j,P_{i}}^{\prime }\right)<f\left(X_{j,Q_{i}}^{\prime }\right),\\ X_{j,P_{i}}^{\prime }+r_{i}\left(X_{j,Q_{i}}^{\prime }-X_{j,P_{i}}^{\prime }\right), & f\left(X_{j,Q_{i}}^{\prime }\right)<f\left(X_{j,P_{i}}^{\prime }\right). \end{array}\right. \end{array}$$

Therefore, the learning phase is modified in conjunction with realistic situations to enhance population diversity and improve the development of algorithms. The modalities are as follows:

(4) $$\begin{array}{c} X_{\text{new}i}=X_{i}+\text{Rand}\left(T_{k}-T_{i}\right). \end{array}$$

*k* is *k* iteration.

*X*_*i*_ is individual.

Rand is random digit.

The instruction is divided into beginner, intermediate, and advanced levels, and students with vocal fundamentals can choose intermediate and advanced levels for their studies [29]. A detailed investigation and careful analysis of user requirements are performed, followed by the development of a unified design specification by designers, domain experts, and knowledge engineers based on the application problem to be solved, specifying the design goals, including the type and scope of the problem itself, and the people involved in the development process. That is, the value of TF decreases linearly as the iterations proceed. The improved teaching factor TF is as follows.

(5) $$\begin{array}{c} \text{TF}={\text{TF}}_{\max}-\left(\frac{{\text{TF}}_{\max}-{\text{TF}}_{\min}}{{\text{iter}}_{\max}}\right)\text{iter} \end{array}$$

TF_max_, TF_min_ are maximum and minimum values of teaching factors.

iter_max_ is maximum iterative algebra.

iter is current iterative algebra.

As a general performing arts discipline, the online vocal classroom is divided into a learner management module, a course education module, and a learning activity module. The online collaborative learning process based on the cloud course platform integrating social media is shown in Figure 2.

Second, by incorporating modern information technology into vocal learning, students can create their own vocal accompaniment using fun software, making their vocal practice more rich and interesting, and by creating their own accompaniment, they can strengthen their inadequate practice and comprehensively improve their vocal level. Under current technical conditions, consult a variety of domestic and international materials to collect, summarize, and organize domain knowledge, select appropriate knowledge acquisition methods, such as manual knowledge acquisition, semi-automatic knowledge acquisition, and automatic knowledge acquisition, and then conceptualize them.

Finally, modern information technology can effectively assist students in recording knowledge points and appropriate practice methods in the classroom, allowing them to practice correctly outside of class time and increasing learning continuity. To align with the characteristics of the problem to be solved, knowledge engineers must collect and reorganize formal knowledge, including the separation of knowledge and fact bases, knowledge representation, implementation of reasoning mechanisms, and human-computer interaction. Based on a thorough understanding of information users' needs, organize digital and web-based information and provide retrieval and relevant links. The most cutting-edge knowledge is delivered to those who need it most, ensuring that information resources are widely disseminated and resources are shared quickly and efficiently. Teachers can share their production results and exchange teaching methods and means via the campus network, which not only improves the quality of teaching but also creates opportunities for new “blood” to enter the teaching circle.

### 3.2. Optimizing Vocal Music Singing with Intelligent Big Data Technology

In traditional vocal music teaching, heuristic teaching mode is often used, which only abstractly introduces the feelings of daily life into vocal singing and allows students to imagine and comprehend the emotions and singing techniques of the songs by themselves [30]. Moreover, with the adoption of digital technology, there is no need to purchase expensive music equipment or to perform routine maintenance tasks. Educators only need basic computer operation skills and basic music knowledge to perform the most basic teaching tasks. The flowchart of the sight-singing and ear training is shown in Figure 3.

First, students can experience the songs directly through multimedia. Music learners access the learning portfolio by logging into the client, which is generally a learning platform, and then present the learning results to the teacher through human-computer interaction. For example, the traditional teaching model of “Morning in Miaoling” with flowery singing is just imagining the text.

Through the means of information technology, the content of the song can be produced, and the birds in the picture can jump to the rhythm. Students can not only hear the song, but also see the song directly and understand their emotions so they can sing with more enthusiasm. The users of the music teaching system include teachers, students, and system administrators. User information management is the basis of system management, including maintenance, query, and statistics of user information. During the teaching phase, individual students are updated by

(6) $$\begin{array}{c} X_{\text{new}}=X_{\text{old}}+{\text{Difference}-\text{Mean}}_{i}. \end{array}$$

*X*_old_ is individual before update.

*X*_new_ is updated individual.

Secondly, through the application of modern information technology, students can use DV to film their singing process, then watch it afterward to find out the deficiencies, and then correct and improve their singing. The core algorithm model of the interactive music intelligence system uses big data technology algorithm. User queries are done by entering user keywords or combining multiple conditions, for any point *x* on the interval [*a*, *b*]; let its reverse point be *x*^*∗*^, the general reverse point be $\bar{x}$, the probability function of any point on the interval to the optimal solution be *P*(·), and the distance function be *d*(·), then the following conclusion holds

(7) $$\begin{array}{c} P\left(d\left(\bar{x}\right)\right)<d\left(x\right)>\frac{1}{2}. \end{array}$$

When the teacher sings the training, they can choose from a number of templates for students with different voice conditions or different singing problems, explaining the key points and difficulties of the class in a variety of ways. The students watching the training can then choose their own optimal solution among these solutions to apply and improve the effectiveness of the lesson. Suppose that in the *k* th iteration, for some individual student *X*_*i*_=(*x*_1_, *x*_2_, ..., *x*_*D*_), such that *M*_*k*_ is the average score of all students and *T*_*k*_ is the teacher, then

(8) $$\begin{array}{c} M_{k}=\frac{1}{NP}\left(\sum_{i=1}^{NP}X_{i,1},\sum_{i=1}^{NP}X_{i,2},...,\sum_{i=1}^{NP}X_{i,D}\right),\\ T_{k}=\min\left\{f\left(X_{i}\right)|i=1,2,...,NP\right\}. \end{array}$$

Finally, we can teach remotely by means of the Internet, which not only saves teaching costs, but also teaches vocal music to a wider range of students. In order to improve the evaluation of the course itself, the review of the singing training evaluation should be conducted by experts, including educational experts, technologists, psychologists, and vocal teaching experts, in addition to the source network. A matrix of size max − iter × *D* and a vector of 1 × max − iter are to be created to store the optimal individual and the optimal fitness values in each generation, respectively. The final space complexity is obtained as

(9) $$\begin{array}{c} S\left(D\right)=O\left(\left(\max-iter+2\times NP\right)\times D\right). \end{array}$$

That is, the basic maintenance of user information includes user name, user number, user address, etc. This basic information is the basis of the system, and the details of users can be viewed at any time throughout the system. The maintenance of user information includes add, modify, and delete operations. When a new user needs to be included in the charge, the user administrator needs to enter the user's details. This is a teaching method that uses Internet technology to solve the space limitation by teaching online instantly. When *D* takes a large enough value, the effect of lower powers on the time complexity is small and can be neglected, then the time complexity of the basic TLBO can be obtained from the above analysis as

(10) $$\begin{array}{c} T\left(D\right)=O\left(\max-\text{iter}\times 2\times NP\times D\right). \end{array}$$

*D* is dimension.

max − iter is iterations.

*NP* is population size.

The premise of this teaching method is to establish a voice or video chat room through the Internet, and then inform and advertise the chat room ID and the arrangement of video vocal teaching, so that people can learn and communicate online at the agreed time. By inheriting the UserControl class, developers can develop various controls according to their needs, and after creation, they can also be compiled into DLL files for other WPF programs to use.

## 4. Application and Analysis of Big Data Technology in the Optimization of Vocal Singing Training

### 4.1. Uncertainty Reasoning Analysis

In the actual development process of expert systems, the problem solving of expert systems is generally not as rigorous and accurate as that of mathematics and physics and other disciplines. Therefore, the knowledge of domain experts and the information we have to deal with are often uncertain and inaccurate.

First, uncertainty and ignorance are distinguished by introducing a trust function, which satisfies the axiom that is weaker than the probability function. Thus, the probability function is a subset of the trust factor. We specify the travel path and remove the average error and low-pass filter or low-precision approximation of the encoded trajectory curve to extract the smooth path curve. The results are shown in Figure 4.

In the control mode of vocal performance or training, students' live participation is added to achieve the basic interaction between computer and music training and performer-human-computer interaction. Through digital technology and multimedia means, animated effects of chest breathing, abdominal breathing, and combined chest and abdominal breathing are created to show the muscle groups in each movement in the working section. It gives the learner an immersive feeling from which he can see why chest and abdominal breathing are not suitable for singing. The multimedia depicts the fuzzy rule count. By learning samples, we try to make the least number of rules to learn and the most important. As the core of digital technology, the computer can be controlled by the teacher. For example, the vocal teacher can control the playing time of the computer music through the pedal, so that the feedback can be used to adjust the teaching at any time, so that the students are really the main focus, using “digital technology” for students and teaching. For the convenience of teachers, some fuzzy quantifiers and quantitative expressions were chosen to represent the confidence level, as shown in Table 1, taking into account the experience of experts in the field.

Second, possibility theory represents uncertainty in terms of likelihood, which is calculated by introducing an affiliation function. Cubase 5 software, developed by Steinberg, was used for the analysis and study. This software not only performs the necessary recording and production functions, but also allows editing the recordings. Another device in this software is a spectrum analyzer, which allows detailed analysis of the singer's spectrum and derives patterns. When targeting a series of larger data, the first *m* of the music data are used as initial training, which leads to the construction of an RBF model of students learning music knowledge, which is continuously evaluated through the designed software platform until a perfect model is finally constructed. Allowing the possibilities of interaction in computer music to be deeper, making this interaction more organic and giving the computer more room to play, for example, allowing the computer to “hear” the singer's real-time vocals or voice while deciding on its own what to feed back. A comparison was made between the performance of the vocal teaching system and the use of computer memory. Figures 5 and 6 compare the CPU and memory usage of the system before and after loading.

Finally, the adequacy and necessity measures are defined as probability ratios, and domain experts are only required to provide probability ratios rather than precise probability estimates. Professional software, on the other hand, can split the singer's voice and accompaniment into two tracks. Following the performance, the tutor can provide a detailed breakdown of what went wrong and improve interactive teaching. The algorithm concept is incorporated into the platform's design, and the algorithm is fully demonstrated while writing the code and implemented in the platform's functions to effectively match the interactive learning mode. By judging the accuracy of the singer's pitch, tone quality, volume, timbre, and vocal language during the singing or vocalization process, the computer determines what, what, how, and how to improve the feedback information. Learners can edit a set of orchestral or band accompaniment tapes to become familiar with the role of each instrument and the combination of accompaniment and voice once they are familiar with the song.

### 4.2. Analysis on the Process of Vocal Music Teaching Optimization

For vocal music teaching, there are certain differences from other teaching. Only very short classroom teaching necessarily requires a strong instantaneous memory, and for some students with weak memories, classroom teaching time becomes insufficient. Such a network means can solve the spatial constraint of the heterogeneous location of vocal learners and vocal teachers, and also allow learners to independently choose their favorite or interested teachers or teaching resources. Therefore, the optimization process of vocal music teaching is as follows.

First, teachers organize exams according to their respective teaching contents, teaching objectives, students' levels and usual exams, log into the system, add exams, select exam topics, receive exam papers, and take exams. The database links between the expert application system and other systems are relatively poor, resource sharing is not fully reflected, unified management is not convenient, and mutual access between users is restricted. All these factors limit the information exchange between expert systems. Therefore, with more and more users of the vocal teaching system, some computer-related hardware indicators such as CPU temperature, CPU package, CPU core difference, and other variables are shown in Figure 7.

However, through intelligent big data technology devices, such as MP4, MD, and some other classical teaching can do “eternal.” On the one hand, after the class, students can listen to what the teacher teaches. On the other hand, teachers can listen to students' classroom recordings to find out some problems of students and develop some targeted measures to solve these problems in the next teaching activities.

Secondly, students choose an exercise mode to practice, and after the diagnostic exercises are completed, the system will analyze the students' exercises according to the exercises.  Figure 8 shows accurately the average response time when different users access the music education information system.

MIDI and ZIPI are the main protocols used in devices to accomplish computer music technology interaction. Therefore, to make a qualitative change in the traditional expert system, the application system of the expert system must first of all have a strong network interconnection function. To achieve network interconnection between expert systems, it is necessary to solve the technical problems of the following kinds of interfaces: the interface between the system and various relational databases, multimedia information processing interfaces, full-text database interfaces, etc. It is a new protocol standard for data exchange between digital musical instruments proposed to overcome many shortcomings such as slow transmission rate and one-way transmission of MIDI. Its transmission rate is nine times that of MIDI, and there is no maximum bandwidth limit in order to adapt to the rapid development of computer technology. In addition, the network media has a huge amount of information, rich information content, and shorter information metabolism cycle, which can enable people to grasp the latest vocal theory knowledge in time and meet their learning needs. The credibility vector is the credibility of the rules in the knowledge base, and the weight vector is the weight vector given by experts. The comparison results of the weight vectors before and after the vocal music teaching optimization process are shown in Table 2.

According to the comparison of the ‘s weight vectors before and after the optimal treatment of vocal music, the weight of the optimal treatment of vocal music increased by 0.154 compared to that before the treatment. Therefore, in this test, the value of the fuzzy term of relative credibility was used; i.e., the credibility was “absolute credibility.”

Finally, a basic evaluation was given after each exercise to encourage students to practice on their own and to pique their interest in learning. This can be done without a tutor at home, at school, anywhere, and at any time. All that is required is that you record the entire process of the tutor's singing using digital multimedia technology, and then record yourself singing and compare the two using the software to see where you went too far in terms of amplitude. The focus on the humanistic aspects of computer music, particularly the interaction of curriculum, vocal training, vocal performance, or lesson production with computer characteristics, can help to establish new computer music aesthetic principles. After all, music intelligence systems are closely linked to teachers, students, and teaching resources, so the corresponding services are slightly different.

## 5. Conclusions

Informationization has already pervaded people's lives, and the information-based classroom will pervade future college classrooms and the general public's learning life. To further improve the shortcomings of traditional vocal teaching methods, existing vocal teaching methods should be combined with digital vocal teaching methods. If multimedia and the Internet are solely used for informational purposes, they will inevitably be phased out over time. Modern information technology, in combination with multimedia and online education, has the potential to significantly improve the quality and efficiency of vocal education, as well as promote vocal singing. Its technical advantages can provide voice learners with a new method of learning vocal art, which has a broad application space and application prospects in the field of vocal education, by optimizing voice training methods based on intelligent big data technology. It completes the basic evaluation of the knowledge points learned by college music teachers and realizes the comprehensive evaluation of a single lesson using a combination of generative and framing knowledge expressions and uncertain reasoning techniques. Vocal music education should not only keep up with the evolution of the information society, but also provide a variety of information services to information users and continue to innovate. The advancement of modern information technology is the general trend, and vocal music must keep up with the times and develop and progress more comprehensively. The combination of big data technology and vocal music education has not only accelerated the diversification of music education, but also improved traditional vocal music education.

## Figures and Tables

**Figure 1:** Interactive learning loop diagram.

**Figure 2:** Design of teaching activities based on network collaborative learning.

**Figure 3:** Flowchart of solfeggio.

**Figure 4:** Results of editing motion path and removing average error.

**Figure 5:** CPU usage comparison.

**Figure 6:** Comparison of memory usage.

**Figure 7:** Curve changes after the number of users increases.

**Figure 8:** Curve of response time.

**Table 1:** Numerical representation of confidence fuzzy quantifiers.

Fuzzy quantifier	Absolutely credible	Strong credibility	Weak credibility	Untrustworthy
Numerical value	1	0.557	0.429	0.186

**Table 2:** Comparison of weight vectors before and after optimization of vocal music teaching.

Weight vector	*μ*_1_	*μ*_2_	*μ*_3_	*μ*_4_

Preweighting	0.556	0.257	0.461	0.672
After weighting	0.672	0.443	0.572	0.875
Differential value	0.116	0.186	0.111	0.203

## Data Availability

The data used to support the findings of this study are available from the corresponding author upon request.

## References

[1] Muzaffarova S., Khurshid B. (2019). Modern training methods in vocal education[j]. *Culture and Arts of Central Asia*.

[2] Fu W., Liu S., Dai J. (2021). *E-Learning, E-Education, and Online Training*.

[3] Wang X. (2022). Design of vocal music teaching system platform for music majors based on artificial intelligence. *Wireless Communications and Mobile Computing*.

[4] Tanik M. M. (2017). Big data optimization: recent developments and challenges.[J]. *Computing Reviews*.

[5] Chen N., Wen G. (2021). Music composition feasibility using a quality classification model based on artificial intelligence[J]. *Aggression and Violent Behavior*.

[6] Zhou M., Gong T. (2020). Optimization of multimedia computer-aided interaction system of vocal music teaching based on voice recognition. *Computer-Aided Design and Applications*.

[7] Zhang W., Shankar A., Antonidoss A. (2021). Modern art education and teaching based on artificial intelligence[J]. *Journal of Interconnection Networks*.

[8] Xu C. (2019). A big-data oriented recommendation method based on multi-objective optimization. *Knowledge-Based Systems*.

[9] Su G. (2019). Analysis of optimisation method for online education data mining based on big data assessment technology. *International Journal of Continuing Engineering Education and Lifelong Learning*.

[10] Park S.-U. (2019). Keyword analysis of data technology using big data technique. *Journal of Korea Technology Innovation Society*.

[11] Wang L., Zhao T., Zhang Y. (2018). Multi-source integration and storage optimization method for big data of power distribution and utilization[J]. *Gaodianya Jishu/High Voltage Engineering*.

[12] Chang Minho M., 김자현 Z. (2019). Technology and big data in music. *The Korean Journal of Arts Studies*.

[13] Nian L., Wang F. (2017). On the importance of emotional cultivation in vocal music teaching[J]. *International Technology Management*.

[14] Shi Z., Bai Y., Jin X., Wang X., Su T., Kong J. (2022). Deep prediction model based on dual decomposition with entropy and frequency statistics for nonstationary time series. *Entropy*.

[15] Wang J., Zhang X., Xu J. (2022). Blockchain-based information supervision model for rice supply chains[J]. *Computational Intelligence and Neuroscience*.

[16] Medeiros L. F. d., Junior A. K., Moser A. (2021). Uma inteligência artificial ensinando sobre inteligência artificial: relato de experiência/an artificial intelligence teaching on artificial intelligence: experience report. *Brazilian Journal of Development*.

[17] Baker V. D., Cohen N. (2017). University vocal training and vocal health of music educators and music therapists.[J]. *Update Applications of Research in Music Education*.

[18] Xiong W., Huang D., Xu W. (2021). Big data and deep learning model for FMS score prediction of aerobics athletes. *Scientific Programming*.

[19] Li Z. (2017). Design of online vocal music course based on Azure-PaaS platform[J]. *International Journal of Emerging Technologies in Learning (iJET)*.

[20] Chi X. (2017). Study on vocal music teaching innovation mode based on computer simulation and voice spectrogram analysis[J]. *Revista de la Facultad de Ingenieria*.

[21] Yang Y. (2020). Application of multimedia technology in vocal music digital teaching reform. *Journal of Physics: Conference Series*.

[22] Rosenzweig S., Scherbaum F., Shugliashvili D., Arifi-Müller V., Müller M. (2020). Erkomaishvili dataset: a curated corpus of traditional Georgian vocal music for computational musicology. *Transactions of the International Society for Music Information Retrieval*.

[23] Simones L. L. . (2017). A framework for studying teachers’ hand gestures in instrumental asnd vocal music context[J]. *Musicae Scientiae*.

[24] Sun Z. (2020). Analysis of the inheritance of traditional music culture based on big data auxiliary technology. *Journal of Physics: Conference Series*.

[25] Sturtevant N. R. (2018). AI education matters. *AI Matters*.

[26] Kim A., Lee J., Kim M. A Study on Music Distribution Framework Using Music Representation Model[C]//.

[27] Du X. (2020). Application of deep learning and artificial intelligence algorithm in multimedia music teaching[J]. *Journal of Intelligent and Fuzzy Systems*.

[28] Zhao M., Jha A., Liu Q. (2021). Faster Mean-shift: GPU-accelerated clustering for cosine embedding-based cell segmentation and tracking. *Medical Image Analysis*.

[29] Sun J. (2019). Research on the reform of information disclosure system of minority college students music education in the age of big data[J]. *Guizhou Ethnic Studies*.

[30] (2021). Research on the reform of vocal music teaching by computer multimedia technology[J]. *Journal of Physics: Conference Series*.

